# FAM83H-AS1/miR-485-5p/MEF2D axis facilitates proliferation, migration and invasion of hepatocellular carcinoma cells

**DOI:** 10.1186/s12885-021-08923-0

**Published:** 2021-12-07

**Authors:** Wenpeng Zhao, Jiang Guo, Honglu Li, Liang Cai, Youjia Duan, Xiaopu Hou, Zhenying Diao, Xihong Shao, Hongliu Du, Changqing Li

**Affiliations:** Department of Oncology Interventional Radiology, Beijing Ditan Hospital, Capital Medical University, No.8 Jingshundong Road, Beijing, 100015 China

**Keywords:** FAM83H-AS1, miR-485-5p, MEF2D, HCC

## Abstract

**Background:**

Abundant evidence has manifested that long noncoding RNAs (lncRNAs) are closely implicated in human cancers, including hepatocellular carcinoma (HCC). Remarkably, lncRNA FAM83H antisense RNA 1 (FAM83H-AS1) has been reported to be a tumor-propeller in multiple cancers. However, its effect on HCC progression remains unknown.

**Methods:**

FAM83H-AS1 expression was analyzed by RT-qPCR. Colony formation, EdU, and flow cytometry as well as transwell assays were implemented to analyze the biological functions of FAM83H-AS1 on HCC progression. Luciferase reporter, RIP and RNA pull-down assays were implemented to detect the interaction among FAM83H-AS1, microRNA-485-5p (miR-485-5p), and myocyte enhancer factor 2D (MEF2D) in HCC cells.

**Results:**

FAM83H-AS1 expression in HCC cells was markedly elevated. FAM83H-AS1 accelerated cell proliferation, migration and invasion whereas inhibiting cell apoptosis in HCC. Besides, we confirmed that FAM83H-AS1 acts as a miR-485-5p sponge in HCC cells. Additionally, MEF2D was verified to be a direct target of miR-485-5p. FAM83H-AS1 could upregulate MEF2D expression via sponging miR-485-5p. Further, rescue experiments testified that MEF2D upregulation or miR-485-5p downregulation offset the repressive effect of FAM83H-AS1 depletion on HCC cell progression.

**Conclusions:**

FAM83H-AS1 facilitates HCC malignant progression via targeting miR-485-5p/MEF2D axis, suggesting that FAM83H-AS1 may be a promising biomarker for HCC treatment in the future.

**Supplementary Information:**

The online version contains supplementary material available at 10.1186/s12885-021-08923-0.

## Background

Diagnosed as the most frequent type of malignancy in men under 60 years old, hepatocellular carcinoma (HCC) accounts for a large proportion of cancer-related deaths all around the world, resulting in no less than 600,000 deaths each year [1–3]. Besides, its incidence rate is approximately equivalent to its mortality rate, indicating that this malignant disease possesses an aggressive nature [4–6]. People chronically infected with the hepatitis B or C viruses and long exposed to dietary aflatoxin B are inclined to suffer from HCC. Additionally, long-term excessive drinking is also a major risk factor of HCC [5, 6]. Multiple therapeutic methods have been explored and implemented to treat HCC over the past years, such as surgical resection, chemotherapy as well as radiotherapy. However, most HCC patients are diagnosed at advanced stages because of lacking effective techniques of early-stage detection, leading to the inapplicability of liver transplantation or surgical resection. Improvements in HCC prevention, intervention, diagnosis and treatment remain limited and unsatisfactory [7–9]. As a result, a penetrated investigation on the underlying molecular mechanism of HCC progression is still the priority for identifying potential biomarkers to develop effective strategies for HCC treatment.

Encoded from mammalian genome, numerous lncRNAs are functionally identified as transcripts with a length of over 200 nucleotides, exhibiting no or limited protein-coding capacity due to a lack of an open reading frame [10, 11]. As documented, lncRNAs are crucial meditators of tumorigenesis by exerting biological functions and inducing regulatory mechanisms in multiple human cancers [12]. Among the regulatory mechanisms, competing endogenous RNA (ceRNA) network is the most prevalent in regulating cellular behaviors of diverse malignancies, including HCC. For example, HIF1A-AS2 propels the progression of colorectal cancer via the regulatory axis of miR-129-5p/DNMT3A [13]. In osteosarcoma, TUG1 motivates cell proliferation whereas represses cell apoptosis by targeting miR-212–3p/FOXA1 axis [14]. In HCC, Unigene56159 positively regulates Slug expression to promote cell epithelial-mesenchymal transition via sponging miR-140-5p [15]. FAM83H-AS1 has been recently verified to accelerate the progression of bladder cancer and glioma [16, 17]. Intriguingly, the facilitating role of FAM83H-AS1 on malignant cellular behaviors in HCC by Wnt/β-catenin pathway has been reported in the previous study [18]. Herein, we further investigated the other regulatory mechanism of FAM83H-AS1 in HCC in terms of ceRNA network.

In conclusion, our study intended to explore the underlying mechanism of FAM83H-AS1 in the progression of HCC, aiming to provide novel insights into HCC treatment.

## Methods

### Cell lines

Human HCC cell lines include Huh7, HepG2, MHCC-97H, and HCCLM3. Huh cell line (CBP30045L; Cobioer, Nanjing, China), MHCC-97H cell line (CBP60227, Cobioer) and normal liver epithelial cell line THLE-3 (CRL-11233; ATCC, Manassas, VA) were all purchased in December, 2019. HCCLM3 cell line (CBP60654, Cobioer) and HepG2 cell line (HB-8065, ATCC) were commercially acquired in April, 2020 and May, 2020 respectively. For cell culture, cells were kept in the DMEM (Invitrogen, Carlsbad, CA) added with 10% FBS and 1% antibiotics. All the above cell lines have been recently authenticated using STR analysis and have been recently tested for no mycoplasma contamination. Cell cultivation was performed in a humidified atmosphere with 5% CO_2_ at 37 °C.

### RT-qPCR

Total RNAs were isolated from HCCLM3 and MHCC-97H cells by TRIzol (Thermo Fisher Scientific, Waltham, MA). Afterwards, reverse transcription of RNAs into complementary DNA (cDNA) was completed using Reverse Transcription Kit (Takara, Otsu, Japan) as the supplier’s manual. QPCR was implemented for quantification of RNA expression with Power SYBR Green (Takara). Target RNA expression was analyzed by 2^−ΔΔCT^ method, standardized to U6 or GAPDH.

### Transfection

HCCLM3 and MHCC-97H cells were inoculated into the 6-well plates for transfection via Lipofectamine 2000 (Invitrogen) for 48 h. The FAM83H-AS1-specific short hairpin RNAs (shRNAs), corresponding nonspecific negative control (NC) of shRNAs (sh-NC), and empty pcDNA3.1 vectors as well as pcDNA3.1/MEF2D, were all commercially obtained from GeneCopoecia (Guangzhou, China). Additionally, miR-485-5p mimics/inhibitor and negative controls NC mimics/inhibitor were all procured from RiboBio (Guangzhou, China).

### Cell proliferation assays

Colony formation and EdU assays were performed to determine cell proliferation. For colony formation assay, transfected HCC cells were seeded into the medium plates (3 × 10^3^/100 μL) with 5% CO_2_ at 37 °C, followed by the incubation for 2 weeks. After rinsing in phosphate-buffered saline (PBS), colonies were fixed and subsequently dyed by 1 mL of 0.1% crystal violet. The colony was defined as a cluster of > 50 cells and colonies were counted manually. For EdU assay, the transfected HCC cells were subjected to EdU assay kit from RiboBio in the 96-well plates as per the instructions of the manufacturer. Cells were visualized under a fluorescent microscope at 20× magnification (Leica, Wetzlar, Germany) after nuclear counterstain with DAPI.

### Flow cytometry analysis

Flow cytometry assay was implemented by utilizing FITC Annexin V Apoptosis Kit (BD Biosciences, San Jose, CA, USA) in line with the guide book. Transfected HCC cells were washed in pre-cooled PBS after trypsin treatment. 5 × 10^5^ cells were cultured in 1 × binding buffer (100 μL) supplemented with PI (5 μL) and FITC Annexin V (5 μL) at room temperature, followed by analysis using a flow cytometer (BD Biosciences).

### Transwell assay

Migration of cells was measured with no-Matrigel-coated transwell inserts while invasion was assessed by use of Matrigel pre-coated transwell inserts (Corning Co., Corning, NY). 5 × 10^3^ cells were paved in the upper chambers of inserts with serum-free medium while the lower chambers were filled with conditioned medium. Subsequent to being fixed, cells migrated or invaded to the lower chambers were dyed by crystal violet for counting by microscopy at 10× magnification.

### Subcellular fractionation assay

For this assay, PARIS™ Kit (Ambion, Austin, TX) was used following the supplier’s instruction. After RNA extraction, the nuclear and cytoplasmic expression levels of FAM83H-AS1 were assayed by RT-qPCR, relative to GAPDH and U6.

### Dual-luciferase reporter assay

FAM83H-AS1 cDNA sequence containing the putative miR-485-5p binding sites was inserted into pmirGLO vectors (Promega, Madison, WI) for the construction of FAM83H-AS1-WT (wild-type) vector. The construct FAM83H-AS1-Mut (mutant) was inserted with the mutant FAM83H-AS1 which contains the mutated seed region binding sites of miR-485-5p. After the co-transfection of the indicated plasmids into cells, luciferase activity was detected via Dual-Luciferase Reporter Assay System (Promega). Firefly luciferase activity was relative to that of Renilla luciferase gene.

### RIP assay

RIP assay was achieved with the help of Magna RIP Kit (EMD Millipore, Billerica, MA, USA) using human Argonaute2 (Ago2) antibodies (anti-Ago2). Magnetic beads were incubated with the indicated antibodies. Cells were lysed in RIP lysis buffer. Cell lysates were acquired for incubation with magnetic beads bound to the indicated antibodies. RNAs were purified from the precipitates and analyzed by RT-qPCR.

### RNA pull-down assay

The sequences of miR-485-5p covering the putative mRNA binding sites were obtained and biotinylated, forming Bio-miR-485-5p. Bio-NC was used as a negative control. The lysates of HCC cells were prepared for the following steps. Magnetic beads were added to the lysates for 1 h. RT-qPCR analyses were finally used for analyzing the enrichment of RNAs in the pull-downed complexes.

### Statistical analysis

Each experiment contained 3 independent bio-repeats, each of which included 3 technical replicates. Results were all shown as mean ± standard deviation (SD). Group comparison analysis was carried out with Student’s t test or one-way/two-way analysis of variance (ANOVA) using Prism 5.0 software (GraphPad Software, Inc., La Jolla, CA, USA), with *p*-value (< 0.05) indicating the statistical difference.

## Results

### FAM83H-AS1 is expressed at high levels in HCC cell lines and promotes HCC cell progression

Recent studies have revealed an obvious elevation of FAM83H-AS1 expression in multiple cancers, including bladder cancer and glioma [16, 17], yet the level of FAM83H-AS1 in HCC remains unknown. Therefore, we applied RT-qPCR to examine FAM83H-AS1 expression and observed a markedly higher expression of FAM83H-AS1 in HCC cell lines (HepG2, Huh7, MHCC-97H and HCCLM3), particularly in the latter two (Fig. 1A). Hence, they were chosen to be used in the subsequent experiments. After the ablation of FAM83H-AS1 by transfection with sh-FAM83H-AS1#1/2 (Fig. 1B), cell proliferative capability was significantly attenuated (Fig. S1A-B, Fig. 1C-D). On the contrary, cell apoptosis was observably enhanced after the depletion of FAM83H-AS1 (Fig. S1C, Fig. 1E). In addition, the migratory capacity and invasive ability of HCC cells were notably impeded by the downregulation of FAM83H-AS1 expression according to transwell assay (Fig. S1D, Fig. 1F). Therefore, it was concluded that FAM83H-AS1 represses cell growth, migration and invasion in HCC.

**Fig. 1:** FAM83H-AS1 is expressed at high levels in HCC cell lines and promotes HCC cell progression. (**A**) FAM83H-AS1 expression in HCC cell lines (HepG2, Huh7, MHCC-97H and HCCLM3) and normal human liver epithelial cell line (THLE-3) was measured by RT-qPCR analysis. (**B**) The knockdown efficiency of FAM83H-AS1#1/2 in HCCLM3 and MHCC-97H cells was detected via RT-qPCR. (**C**-**D**) The proliferation ability of HCC cells transfected with downregulated FAM83H-AS1 was assessed via colony formation and EdU assays. (**E**) Flow cytometry analysis was conducted to determine the apoptosis of HCC cells before or after the silencing of FAM83H-AS1. (**F**) The migratory and invasive abilities of transfected cells were evaluated via transwell assays. ^**^P < 0.01. See related supplementary data in Fig. S1 and S2

Besides, we further demonstrated the gain-of-function effects of FAM83H-AS1 on HCC progression. Firstly, we testified the upregulation efficiency of pcDNA3.1/FAM83H-AS1 before gain-of-function experiments (Fig. S2A). Upregulated expression of FAM83H-AS1 markedly increased colony number and rate of EdU positive cells (Fig. S2B-C). High expression of FAM83H-AS1 led to the decreased apoptotic rate of HCC cells (Fig. S2D). As for the migratory and invasive capacities, transwell assays showed that number of both migrated and invaded cells was significantly improved (Fig. S2E). Taken together, FAM83H-AS1 expression in HCC cells is significantly upregulated and knockdown of FAM83H-AS1 has the inhibitory effect while FAM83H-AS1 overexpression has the opposite effect on HCC cell progression.

### FAM83H-AS1 targets miR-485-5p directly in HCC cells

To decipher the underlying mechanism of FAM83H-AS1 in HCC cells, we preliminarily performed cytoplasmic-nuclear fractionation assay and discovered that FAM83H-AS1 was largely localized in the cytoplasm of HCCLM3 and MHCC-97H cells (Fig. 2A). Thereby, we boldly raised a speculation that cytoplasm-distributed FAM83H-AS1 probably acts as a ceRNA. Through the prediction of lncRNASNP2 database and DIANA tools, 6 microRNAs (miRNAs) were predicted to combine with FAM83H-AS1 (Fig. 2B-C). To identify the specific downstream miRNA of FAM83H-AS1 in HCC cells, RT-qPCR assay was carried out. The results delineated that only miR-485-5p was remarkably lowexpressed in HCC cells (Fig. 2D). After the downregulation of FAM83H-AS1 expression, miR-485-5p expression was conspicuously upregulated in HCC cell lines relative to THLE-3 cell line (Fig. 2E). Successively, the binding site of FAM83H-AS1 with miR-485-5p was obtained via lncRNASNP2 prediction (Fig. 2F). Later on, we found that overexpressing miR-485-5p (Fig. 2G) distinctly reduced the luciferase activity of FAM83H-AS1-WT whereas that of FAM83H-AS1-Mut had no significant change (Fig. 2H). Finally, RIP assay was carried out to determine the interaction probability of FAM83H-AS1 with miR-485-5p. Results manifested that FAM83H-AS1 and miR-485-5p were both much enriched in anti-Ago2 groups relative to those in anti-IgG groups (Fig. 2I). As Ago2 is an essential component of RISCs (RNA-induced silencing complexes), the results proved the co-existence of FAM83H-AS1 and miR-485-5p in RISCs [19]. To conclude, FAM83H-AS1 binds to miR-485-5p in HCC cells.

**Fig. 2:** FAM83H-AS1 directly targets miR-485-5p in HCC cells. (**A**) The location of FAM83H-AS1 in HCC cells was detected. (**B**-**C**) 6 candidate miRNAs were predicted to bind to FAM83H-AS1 through the combined analysis of lncRNASNP2 database (http://bioinfo.life.hust.edu.cn/lncRNASNP#!/) and DIANA tools (http://carolina.imis.athena-innovation.gr/diana_tools/web/index.php?r=lncbasev2/index-predicted). (**D**) The expression of these candidate miRNAs in HCC cells and THLE-3 cells was evaluated via RT-qPCR analysis. (**E**) Detection of miR-485-5p expression was performed via RT-qPCR analysis in FAM83H-AS1-depleted HCC cells. (**F**) The potential binding site between FAM83H-AS1 and miR-485-5p predicted by lncRNASNP2 was shown. (**G**) RT-qPCR was applied to validate the upregulation efficiency of miR-485-5p. (**H**) The luciferase activity of FAM83H-AS1-WT/Mut was detected in miR-485-5p-overexpressed HCC cells. (**I**) The enrichment of FAM83H-AS1 or miR-485-5p in Anti-Ago2 bound precipitates was detected in RIP assays. ^*^P < 0.05, ^**^P < 0.01

### FAM83H-AS1 indirectly regulates MEF2D expression in HCC cells

To further probe into the potential ceRNA mode of FAM83H-AS1 in HCC cells, we employed miRWalk database to speculate downstream targets of miR-485-5p. As illustrated in Fig. S3A, 10 putative mRNAs were predicted to combine with miR-485-5p. RNA pull-down assay displayed that only MEF2D presented an evident abundance in bio-miR-485-5p groups, manifesting the binding potential between miR-485-5p and MEF2D in HCC cells (Fig. 3A). Furthermore, either miR-485-5p upregulation or FAM83H-AS1 downregulation could cut down the expression of MEF2D in HCC cells (Fig. 3B-C). Besides, RT-qPCR analyses revealed a significant elevation of MEF2D expression in HCC cells in comparison with that in THLE-3 cells (Fig. 3D). The binding site between MEF2D and miR-485-5p was obtained by TargetScan prediction (Fig. S3B). After the upregulation of MEF2D expression (Fig. 3E), the repression of luciferase activity of FAM83H-AS1-WT caused by miR-485-5p overexpression was counteracted while luciferase activity of FAM83H-AS1-Mut had no marked change (Fig. 3F). After transfection of miR-485-5p inhibitor, the level of miR-485-5p was obviously decreased in HCC cells (Fig. 3G). Further, the impaired expression of MEF2D induced by FAM83H-AS1 knockdown could be rescued via inhibiting miR-485-5p expression or overexpressing MEF2D (Fig. 3H). To sum up, FAM83H-AS1 regulates MEF2D expression by sponging miR-485-5p.

**Fig. 3:** FAM83H-AS1 indirectly regulates MEF2D expression in HCC cells. (**A**) The binding ability of miR-485-5p with candidate mRNAs was tested via RNA pull-down assay. (**B**-**C**) MEF2D expression in different transfected cells was measured via RT-qPCR analysis. (**D**) MEF2D expression in HCC cell lines and THLE-3 cell line was examined by RT-qPCR analysis. (**E**) Evaluation of MEF2D overexpression efficiency was conducted via RT-qPCR. (**F**) The luciferase activity of FAM83H-AS1, miR-485-5p or MEF2D was detected in the indicated transfected HCC cells. (**G**) The inhibition efficiency of miR-485-5p inhibitor was verified via RT-qPCR. (**H**) MEF2D expression in different groups was examined by RT-qPCR analysis. ^**^P < 0.01

### FAM83H-AS1 enhances the progression of HCC cells via miR-485-5p/MEF2D axis

To further testify whether FAM83H-AS1 contributes to HCC cell progression by regulating miR-485-5p/MEF2D axis, rescue assays were performed successively. Colony formation and EdU assays uncovered that miR-485-5p ablation or MEF2D upregulation could counteract the repressive impact of FAM83H-AS1 silence on cell proliferation (Fig. S4A-B, Fig. 4A-B). In addition, cell apoptosis ability facilitated by inhibited FAM83H-AS1 was counteracted by miR-485-5p suppression or MEF2D upregulation (Fig. S4C, Fig. 4C). Furthermore, through transwell assay, we discovered that miR-485-5p silencing or MEF2D upregulation countervailed the inhibitory influence of silenced FAM83H-AS1 on HCC cell migration and invasion (Fig. S4D, Fig. 4D). In sum, FAM83H-AS1 elevates MEF2D expression to facilitate HCC cell proliferation, migration and invasion by sponging miR-485-5p (Fig. S5).

**Fig. 4:** FAM83H-AS1 motivates the malignant progression of HCC cells via miR-485-5p/MEF2D axis. (**A**-**B**) The proliferation ability of transfected HCC cells was assessed by colony formation and EdU assays. (**C**) Flow cytometry analysis was performed to examine the apoptosis of transfected cells. (**D**) The migratory and invasive capabilities of HCC cells in different groups were evaluated via transwell assays. ^**^P < 0.01. See related supplementary data in Fig. S4

## Discussion

Accumulating cancer-related studies have manifested the cancer-facilitating or restraining roles of abnormally expressed lncRNAs in a string of biological processes of HCC cells. For instance, lncRNA CCAT1 drives HCC cell proliferation and migration by sponging let-7 [20]. Elevated expression of lncRNA ZEB1-AS1 promotes HCC progression and indicates poor prognosis [21]. LncRNA NEAT1, acting as a ceRNA, facilitates HCC development by regulating miR-485/STAT3 axis [22]. Although FAM83H-AS1 has been revealed to facilitate the incidence and development of bladder cancer and glioma [16, 17], the studies on the underlying effect of FAM83H-AS1 on HCC are exceedingly limited. Based on the previous studies, we found that FAM83H-AS1 in HCC tissue samples is highly expressed compared with that in non-tumor tissue samples (^*^P < 0.05), and positively correlated with HCC tumor size and vascular invasion [18]. Consistently, the present study discovered the dramatically upregulated FAM83H-AS1 in HCC cells. Elevation of FAM83H-AS1 expression was found to promote the proliferative, migratory and invasive capacities while inhibiting the apoptosis of HCC cells, which is in accord with the finding reported in the previous study [18].

Defined as a class of small noncoding RNA molecules with less than 25 nucleotides at length, miRNAs have been widely uncovered to serve as significant participators in various cellular processes in cancer, such as cell proliferation, apoptosis and migration [23–25]. Existing studies have revealed that lncRNAs may elicit pivotal effects on the development and progression of human cancers (HCC included) via regulating certain miRNA [26–28]. In this study, we originally detected that FAM83H-AS1 was largely distributed in the cytoplasm of HCC cells and accordingly, we boldly speculated that FAM83H-AS1 probably might serve as a ceRNA of a specific miRNA. Although miR-485-5p has been depicted as an anti-tumor gene, and was expressed at low levels in HCC tissues [29], the function that the interaction between FAM83H-AS1 and miR-485-5p exerts on HCC development still requires in-depth investigation. Through bioinformatics prediction and mechanism experiments, we validated that FAM83H-AS1 binds to miR-485-5p and serves as a negative regulator of miR-485-5p expression.

According to the existing literatures, signally elevated expression of MEF2D has been unveiled in several human cancers and MEF2D upregulation contributes to the development of cancers, such as pancreatic cancer [30] and lung cancer [31]. In our study, we found that MEF2D expression was significantly increased in HCC cell lines, being in line with its upregulation in HCC tissues [32]. In this investigation, MEF2D was verified to be a target of miR-485-5p in HCC. More importantly, through rescue assays, we certified that FAM83H-AS1 could elevate MEF2D expression through sponging miR-485-5p. Further, either upregulating MEF2D expression or inhibiting miR-485-5p expression could offset the suppression on HCC progression caused by FAM83H-AS1 downregulation.

## Conclusion

To sum up, FAM83H-AS1 facilitates HCC progression by targeting miR-485-5p/MEF2D axis. This finding provides evidence of FAM83H-AS1 as an oncogene along with its ceRNA mechanism in HCC, shedding light on developing therapeutic approaches for HCC patients.

## Supplementary Information

**Additional file 1: Fig. S1.** (A-D) Representative images of Fig. 1C-F were shown.

**Additional file 2: Fig. S2.** (A) RT-qPCR analysis was used to verify the overexpression efficiency of pcDNA3.1/FAM83H-AS1 in transfected HCCLM3 and MHCC-97H cells. (B-C) The proliferation of FAM83H-AS1-overexpressed HCC cells was assessed by colony formation and EdU assays. (D) Flow cytometry analysis was carried out to detect the apoptosis of HCC cells before or after the overexpression of FAM83H-AS1. (E) Transwell assays were implemented to evaluate the migratory and invasive capacities of pcDNA3.1/FAM83H-AS1-transfected cells. ^**^P < 0.01.

**Additional file 3: Fig. S3.** (A) 10 potential mRNAs which combine with miR-485-5p were predicted through miRWalk database analysis (http://mirwalk.umm.uni-heidelberg.de/). (B) TargetScan database (http://www.targetscan.org/vert_72/) predicted the binding site between MEF2D and miR-485-5p.)

**Additional file 4: Fig. S4.** (A-D) Representative images of Fig. 4A-D were shown.

**Additional file 5: Fig. S5.** The schematic image drawn by the authors presented that FAM83H-AS1/miR-485-5p/MEF2D axis facilitates proliferation, migration and invasion of HCC cells.

## Data Availability

The datasets used and/or analysed during the current study are available from the corresponding author on reasonable request.

## Abbreviations

lncRNAs: long noncoding RNAs
HCC: hepatocellular carcinoma
FAM83H-AS1: FAM83H antisense RNA 1
MEF2D: myocyte enhancer factor 2D
ceRNA: competing endogenous RNA
cDNA: complementary DNA
NC: negative control
PBS: phosphate-buffered saline
WT: wild-type
Mut: mutant
SD: standard deviation.
miRNAs: microRNAs
RISCs: RNA-induced silencing complexes
